# Study of the Effectiveness of 5G Mobile Internet Technology to Promote the Reform of English Teaching in the Universities and Colleges

**DOI:** 10.1155/2022/3053694

**Published:** 2022-07-13

**Authors:** Zhiyong Hu

**Affiliations:** Department of Foreign Language and Tourism, Hebei Petroleum University of Technology, Chengde 067000, Hebei, China

## Abstract

The development of educational information processes and information technology has made it possible to build a remote learning environment for English education. The application of fifth-generation communication (5G) has carried out revolutions in education for both teachers and students. In this study, an optimization approach is presented for English teaching mode to overcome the limits of current college English teaching settings and broaden the span of 5G technology. The proposed optimization technique varies from traditional college English teaching methods in that it integrates 5G, which considerably increases the communication of college English classes. Furthermore, the optimization technique can promote the standard of English teaching in several ways while completely and systematically following the teaching principle of “teach students according to their capabilities.” In addition, a Bat Optimization Algorithm (BOA) is employed to enhance the process of transmission and measure the students' cognitive skills. The experimental results show that the proposed method addresses the limitations of the traditional English teaching model in colleges while enhancing students' cognitive skills in a variety of areas, including listening, speaking, reading, and writing.

## 1. Introduction

Smart classroom technology is helpful in lecture halls and classrooms. By incorporating current technology, these rooms provide learning and instructional opportunities as well as networking and multimedia capabilities [1]. Presentation, administration, accessibility, real-time interactions, and analysis may all be summed up in the acronym “SMART.” The qualities of a “SMART” conceptual model include all the functions of a smart classroom [2]. Learners' motivation may be increased, and their speaking abilities can be improved by integrating 5G and English education to build a new model of teaching the English language [3]. Artificial Intelligence (AI) and 5G are two possibilities for the creation of more advanced educational communications systems. Machine learning, convolutional neural networks, and reinforcement learning are all emerging technologies with a lot of promise in terms of producing highly effective teaching and learning systems. As one of the most important study goals in second-language acquisition, English learner motivation has long been a research issue [4].

With the development of 5G communication networks, online English courses as well as modifications in inspiration to study have received increased devotion from people from all walks of life [5]. However, research outcomes on enthusiasm in conventional foreign language classrooms are hard to adjust to the online English learning environment, and as a result, the number of inducements available to online second language learners has declined [6]. Traditional static inspiration theory cannot be used to explain and examine dynamic change. As a consequence, the matter of discouragement among students enrolled in online English courses via distance education has swiftly emerged as a new subject in second language studies [7]. It is essential to create a 5G wireless distance English learning system of mobile edge computing to improve student comprehension and boost student and teacher interaction while also enabling students and instructors to connect and study with one another regardless of time or place [8]. As a consequence of educational reform, a considerable effect on the area of education in modern society has been created. Modifications in educational institutions are affecting students' intellectual skills, learning processes, interpersonal connections, and self-evaluation [9]. Students may be able to study more intelligently in the 5 G-based education environment supported by mobile computing technologies.

Although earlier research can help better understand online education, the experimental results are not always constant. The sample sizes in those studies are small, and the conclusions are not widely accepted. In this study, a computational analytic approach and a questionnaire survey method based on 5G are used to construct a unique evaluation system comprised of college teachers and students. To successfully deliver instructional content to the receiver, an energy-efficient lecture transmitting technique is used. To maximize transmission, a Bat Optimization Algorithm (BOA) is employed. Results are generated to measure the student's cognitive skills. The study also highlights the current obstacles in English teaching and provides solutions, which will assist in the enrichment of online teaching materials and the development of college instructors' teaching quality.

The rest of the manuscript is organized as follows: Section 2 provides a comprehensive analysis of the related works. In Section 3, a detailed illustration of the proposed method is presented. The results are explained in Section 4, and Section 5 concludes the manuscript.

## 2. Related Works

To enhance the school's overall teaching quality assessment system, it is critical to build a perfect classroom teaching quality evaluation system and conduct frequent objective, fair, and scientific assessments of instructors' teaching effectiveness. To create such a system, Cheng et al. [10] combined the B/S design pattern with the SSM architecture and database development. The system's principal task is to assess the students getting the quality of education provided by course teachers online. Xu [11] employed mobile learning and smartphones to provide an overview of the concept and features of mobile learning and cell phones as well as the supporting theory and technology provision for mobile learning. Furthermore, because of the expansion of mobile Internet, an innovative technique of English training was developed. Zhang and Bi [12] added to the theoretical foundations and practical applications of mobile learning.

A computer-aided design (CAD) theoretical model may help to popularize mobile learning in English while also enhancing teaching quality. Jiao [13] used an edge-based mobile paradigm for learning the English language. Edge computing and network architecture were incorporated because of cognitive flexibility theory and informal learning theory as well as situational network and cognition framework. A mobile English teaching model was proposed based on “listening, reading, and hearing.” Huang and Mai [14] created a learner and teacher-centered model, incorporated a suspicious degree upgrade model into the interest model, and used a machine learning technique called deep learning network algorithm to offer composition resources and achieve composition resource recommendation accuracy. Furthermore, based on real-world requirements, a system structure is presented that determines each of its functional modules' implementation. Chen [15] increased students' performance by using English writing and communication technologies based on 5G networks. The author in [16] adopted a dynamic form of mechanical manufacturing instruction inside a network teaching environment. They studied essential subjects such as the technique for creating a virtual network platform and the operating principles of virtual reality technology before defining the critical technology for a network teaching environment. Chen and Wang [17] explained how network multimedia courseware may be used in college basketball education. They begin by developing a multimedia courseware teaching plan that includes teacher supervision, student learning, and multimedia instructional materials. Second, the Flash mx2004 plug-in was used to complete course contents of multimedia teaching basketball fundamentals. Mo and Yan [18] looked into how higher professional college students can expand their abilities to study English independently, with an emphasis on informatization, to stimulate bilateral communication between students and teachers, promote students' consciousness of lifetime learning, increase teachers' technical skills, and advance a connotative system in higher professional schools. Dou [19] explores the application of wearable technology and how it might be used to teach English in a college setting. A questionnaire was utilized to collect data from students and teachers in this study. Wearable technology, according to the study's conclusions, may pique students' curiosity in college English. The following study proposes to accomplish an interdisciplinary investigation on multimodal semiotics and human education practices to broaden the field of research and preserve some of the vitality of multimodal discourse analysis.

Teaching English as a second language is hard for anybody, regardless of ability level. In places where English is only used in a limited capacity, teaching and learning the language become much more important and cumbersome. Using 5G mobile internet-based training intends to advance the efficacy of English education in universities while simultaneously improving students' knowledge of other academic fields. A preprint has previously been published at Research Square [20].

## 3. Proposed Methodology

This proposal depicts the overall organization of future English classrooms that will be based on 5G networks communications. The most important step is to look into methods for applying organized and intellectual English education in universities and a smart classroom education atmosphere. The number of intellectual classroom education platforms is predictable to triple in the next five to seven years. Following that, an overview of the requirements analysis, performance assessment, and practical design of the network education system in light of the system's 5G network is presented.  Figure 1 depicts a schematic illustration of the proposed method.

### 3.1. Data Collection

In this study, an English education database was employed. The database is publicly available at https://unimelb.libguides.com/2ndlanguage/databases. For students involved in teaching second languages, the database may be utilized as a research tool.

### 3.2. Data Normalization

The input data may include duplicate packets as well as missing data. Duplicate or redundant data and missing data are usually deleted in the cleaning and preprocessing phase. Because of the large quantity of data in the educational systems, sampling methods are used. In this study, owing to the enormous number of features in this data set, a feature extraction strategy is obligatory to eliminate the qualities that are not required. Normalization is used to bring all the values under a common scale. Therefore, it is essential to normalize the data set [21]. The first stage in the normalizing procedure is to get the z-score, which may be expressed by the following equation:

(1) $$\begin{array}{c} Z=\left[\frac{\text{SDD}}{\left(U-\sigma \;\right)}\right], \end{array}$$

where *α* is the mean and SDD signifies the standard deviation. The *z*-score is computed as

(2) $$\begin{array}{c} Z=\frac{U-\bar{U}}{\text{SDD}}, \end{array}$$

where $\bar{U}$ indicates the mean of the sample.

The random sample selected follows the pattern of

(3) $$\begin{array}{c} Z_{j}=\beta_{0}+\beta_{1}U_{j}+\in_{j}, \end{array}$$

where ∈_*j*_ indicates the errors, relied on the *SSD*^2^. As a result, the errors must be independent of one another, as given in the following equation:

(4) $$\begin{array}{c} U_{j}∼\sqrt{W}\frac{U}{\sqrt{U^{2}+w-1}}, \end{array}$$

where *U* indicates a random variable. The moment scale deviation is estimated with the help of the following equation:

(5) $$\begin{array}{c} M=\frac{\lambda^{m}}{\gamma^{m}}, \end{array}$$

where  *m*  indicates the moment scale.

(6) λm=EU−σ^M,

where *Y* indicates a random variable and *E* signifies the value that is expected.

(7) γm=EU−σ^M^2,

(8) $$\begin{array}{c} y_{w}=\frac{m}{\bar{U}}, \end{array}$$

where *y*_*w*_ implies the coefficient of the variance.

This feature scaling procedure is ended when all the variables are set to 0 or 1 at the same time. This method is known as the Unison-based normalizing approach. The normalized equation will be written as follows:

(9) $$\begin{array}{c} U^{\prime }=\frac{\left(U-U_{\min}\right)}{\left(U_{\max}-U_{\min}\right)}. \end{array}$$

In this manner, the data set may be controlled, and the data's size, as well as variation, can be kept constant. The normalized data are used in the subsequent stages of the project.

### 3.3. 5G Network Implementation

In this study, an investigation is made towards a 5G wireless network design where all sensor nodes (SNs) and gateways are arbitrarily distributed and made fixed after use. The SNs are assigned to each gateway if the sensor nodes' contact is within the gateway's contact range. As a consequence, SNs may be allotted to prefixed gateways. Between sensor nodes, a minimum number of portals are deployed. As a consequence, each SN has its own set of portals to choose from. Data collection is divided into phases in the DSR research plan, but the data collection process is also divided into rounds. Both SNs gather data from the local area after each cycle and transmitted it to the relevant gateway (CH). As a result, the data gates delete obsolete and uncorrelated data before delivering it to the base station (BS), utilizing another CH as a next-hop relay node. After two rounds of shutting off their energy-saving radios, the two nodes detach from the network. Everyone gets access to the Internet through 5G Wi-Fi. Even when two nodes are near together, they are still wirelessly connected.

### 3.4. Optimization-Based Energy-Efficient Routing Protocol (BOABEERP)

Bats leave their colony in search of food, and they follow the prey they come upon. Bats emit pheromones as they fly, leaving a trail of their whereabouts behind them. The concentration of a pheromone along a certain path indicates that it is being used. The concentration of pheromones decreases as time passes due to diffusion processes. This is very normal. This capability is critical to the functioning of path searching due to its dynamic nature. Based on the bat foods search mechanism, the proposed routing mechanism is thoroughly investigated after the establishment of clusters. We go through two phases in this procedure: picking a reliable node and determining the best path. First, depending on other users' trust ratings, the proposed algorithm selects the safest approach. In this case, the node symbolizes a swarm of bats. It is a representation of a bat's flight route that is been made. The wireless environment with fifteen nodes is employed to determine the nodal trust value, with the beginning trust value set to zero. We employed the BOABEERP as a data transmission protocol in our work. The dependability and availability criteria are used to calculate the trust score for each node. Those that legally recognize packets they receive from neighbors by replying to the sender make up the first group of nodes. To determine the trust value, numerous routing factors or routing metrics (such as to request, response, and error, among others) are used (bandwidth, cost, etc.). The node is assigned to Group 2 when a large number of packets are sent out at the same time. The rate of genuine acknowledgment may be computed using the equation once all nodes' input energy levels have been calculated as shown in the following equation:

(10) $$\begin{array}{c} {\text{SR}}_{\left(1,j\right)}=\;\frac{\left[C_{1}\times \left(\left(\text{ACK}/\text{NP}\right)\times 100\right)+C_{2}\times {\text{Temp}}_{\text{score}}C_{3}\times {\text{Spatial}}_{\text{score}}\right]}{\left[C_{1}+C_{2}+C_{3}\right]}, \end{array}$$

where *C*_1_, *C*_2_, and *C*_3_ represent the weights applied to several energy values, TR_(1, *j*)_ signifies the initial energy ratio for the *j*^th^ node, ACK denotes the number of acknowledgments sent to neighbor hosts, and NP represents the number of packets received from neighbor nodes, and TR_(1,*j*)_ is the initial energy ratio of the *j*^th^ node. Equation (2), which estimates the released packet, is used to determine the adjacent nodes' trust score.

(11) $$\begin{array}{c} {\text{SR}}_{\left(2,j\right)}=100-\left(\left(\frac{\text{SRP}}{\text{TSRP}}\right)\times 100\right)\text{t}1<\text{t}<\text{t}2, \end{array}$$

(12) $$\begin{array}{c} {\text{SR}}_{\text{Fitnessvalue}}=\frac{\left({\text{SR}}_{\left(1,j\right)}+{\text{SR}}_{\left(2,j\right)}\right)}{2}+\text{FS}, \end{array}$$

where FS is the fitness score, fitness value refers to the overall nodal trust score, SR_(1,*j*)_ refers to the initial trust score, and SR_(2,*j*)_ refers to the second trust value for node *j*.

where SR_(2,*j*)_ signifies the neighbor trust value ratio for the *j*^th^ node, SR is the packet count unconfined, TSRP denotes the whole packet numbers released in the network, and *t* denotes the temporal constraint to check the time boundaries t1 and t2 for lowest and highest time gap limitations. Finally, using the equation, the total trust value of the route particular node *j* is calculated.

Once the trusted node has been identified, the trusted route may be selected. Consequently, dynamic values are preferable to static ones when it comes to prefixes. We can group the routing events using our approach as the signal intensity of the nodes decreases with distance, *d*, as shown in Figure 1. With the use of equation (13) and the distance between two nodes, the amount of energy necessary to transport *k* bits is computed. Consequently, we feel that dynamic values are preferable to static ones when it comes to prefixes. Using the proposed method, we may group the routing events like bats.

(13) $$\begin{array}{c} En_{tx}\left(k,d\right)=k\times En_{\text{elec}}+k\times \varepsilon \times d^{m}, \end{array}$$

where *En*_*ix*_ is the amount of energy used by the BATS and *En*_elec_ is the amount of energy lost by the broadcasting circuit. Based on multipath fading, *m* gets a value of 2 or 4. The energy required for electrical amplification is represented as *ε*.

The average values of the complete trust values for every BAT node available in the network are computed as

(14) $$\begin{array}{c} {\text{BAT}}_{\text{route}}=\overset{m}{\underset{j=1}{\sum }}\frac{{\text{TR}}_{j}}{m}, \end{array}$$

where BAT_route_ denotes the average route trust value, TR_*j*_ is the trust score collection, and *m* refers to the number of bats. When the data have been recognized, it will be transferred across the trusted route. The data are collected by CH over a cluster route created specifically for the SNs. Finally, the sink node's data may be accessed. Algorithm 1 is illustrated.

## 4. Results and Discussion

In this section, the proposed technique is evaluated. Building an English educational system as a first point is required to conduct in-depth conversations about 5G networks and the 5 G-based educational system. It is essential to create an intelligent classroom education information transmission system for the English information system based on the 5G-education network to operate properly.  Figure 2 depicts the artistic skills ability of students in six classes after the application of 5G communication systems in English learning.

From Figure 2, it can be seen that after analyzing the results, the participants' English ability in listening, speaking, learning, and creative thinking has been improved to a certain level. In comparison to traditional face-to-face learning, the education given over 5G Internet has a much larger effect. Comparing 5G computing-based distance education to conventional teaching methodologies, the latter has double the impact and is 50% more economical.

Figure 3 shows that students' English language skills greatly improve, showing that 5G-based online training may surpass the traditional physically learning strategy. It was found that the overall increase in student performance after 5G-based training was greater than the improvement seen in following physical classes.

Figure 4 illustrates that, before 5G-training, the students' ability to do a variety of language capabilities is not well and even that they are not up to the required standard.

Figure 5 shows that, after 5G-training, students' abilities in a variety of activities have increased significantly, and their academic performance has outperformed their abilities.

Figure 6 provides a comparison of the analysis of the two groups' test scores. The average student results were computed using covariate-adjusted regression for each condition using the final test score, average assessment score, and self-reported student happiness. The final test score for the English 5G-classroom scale with learning level analysis is 80%, the average assessment score is 63%, and the student satisfaction score is 80%, all of which are excellent results.

Figure 7 demonstrates that in smart classrooms, most learners favor the traditional audio transmission strategy; however, 5G English classroom sessions may be advantageous. The questionnaire is designed to elicit student viewpoints on themes such as pleasure, knowledge, organization, and the utility of educational success in English smart classrooms in general as well as the value of educational effectiveness. The replies supplied by interview participants are assessed using the scales listed below: Strongly Agree, Agree, and Undecided, Disagree, and Strongly Disagree. According to the study's findings, learners' perceptions of the usage of smart classroom education are strongly agreed upon by 55%, agreed with by 75%, uncertain by 32%, disagreed upon by 22%, and very disagreed upon by 13%.

Figure 8(a) demonstrates that conventional teaching does not provide high levels of satisfaction, which are much lower than the levels of satisfaction associated with simulated 5G online instruction. A kind of remote learning is simulated in 5G Internet education. Multimedia network teaching is considered to be part of the third generation of distance learning, based on contemporary advances in mass media and information technology. Students find simulated 5G online training especially enticing since it is the product of some breakthroughs in advanced computer networks and multimedia technologies. Several calculation and statistical algorithms were used to compare the expenditures of diverse teaching strategies, and a conclusion was reached after gathering relevant data on the costs of these various types of teaching methods. As a result of the variations in algorithm training, different algorithm implementation results are conceivable. Despite certain discrepancies, the differences in relative performance between different algorithms should be small. Figure 8 depicts the specific details (b). In comparison to other existing methods, the results obtained utilizing the proposed methodology demonstrate that it generates good results.

## 5. Conclusion

Conventional classroom arrangements and internal organization have little to do with digital innovations in the modern educational system. Learning settings, student expectations, educational learning strategies, and resources are all examined and considered in smart classrooms. Smart classrooms will help students who are curious to read, write, investigate, technology, or academics and will benefit from smart classrooms. Implementation and application of this advanced technology in primary schools should drive higher education courses in the current educational system. Students and instructors can acquire new skills and opportunities to study in creative and engaging ways in smart 5G classrooms. Students and instructors can rapidly transition to a technology era and digitalization. Consequently, higher learning engagement will assist students in adapting to varied learning modalities. Students and teachers will always change and improve themselves in and out of the classroom. In this study, an English teaching method based on a smart 5G network is presented. Results showed that 55% of students highly agreed, 75% agreed, 32% were unsure, 22% disagreed, and 13% strongly objected to the usage of smart classroom training.

## Figures and Tables

**Figure 1:** The framework of the proposed method.

**Figure 2:** Artistic skills vs parameter value.

**Figure 3:** Class and parameter value.

**Figure 4:** Class vs parameter values before training.

**Figure 5:** Class vs parameter values before training.

**Figure 6:** Score analysis.

**Figure 7:** Learners level analysis.

**Figure 8:** Comparative analysis.

**Algorithm 1:** 5G_Bat optimization.

## Data Availability

The experimental data used to support the findings of this study are available from the author upon request.
